# Endothelium-dependent and endothelium-independent vasorelaxant effects of unripe *Rubus coreanus* Miq. and *Dendropanax morbiferus* H. Lév. extracts on rat aortic rings

**DOI:** 10.1186/s12906-020-02977-6

**Published:** 2020-06-22

**Authors:** Soyi Park, Ki Hoon Lee, Wan Seok Kang, Jin Seok Kim, Sunoh Kim

**Affiliations:** Central R&D Center, Bioresources and Technology (B&Tech) Co., Ltd., 257, Jebong-ro, Buk-gu, Gwangju, 61239 South Korea

**Keywords:** Unripe *Rubus coreanus* Miq., *Dendropanax morbiferus* H. Lév., Hypertension, _L_-arginine, GABA, Nitric oxide

## Abstract

**Background:**

Many clinical trials on antihypertensive drugs have confirmed the usefulness of these drugs in regulating blood pressure effectively. However, all the drugs usually require long-term use; thus, economic burdens as well as some adverse effects, including headache, diarrhea, skin rash, edema, fever, and liver and kidney dysfunction, accompany their use. Therefore, we attempted to identify natural medications for treating hypertension. We investigated the antihypertensive effects of *Dendropanax morbiferus* H. Lév. extract (*DP*), enzymatically hydrolyzed *DP* extract (Hy-*DP*) and 5% unripe *Rubus coreanus* Miq. ethanol extract (5-*u*RCK).

**Methods:**

Extracts of the unripe *R. coreanus* were made using 20 volumes of 5% ethanol at 100 °C for 4 h. The dried leaves of *D. morbiferus* were subjected to enzymatic hydrolysis by protease, trypsin, bromelain and papain to increase _L_-arginine and GABA levels. Vasorelaxant effects of these extracts were evaluated on rat aorta precontracted with phenylephrine. In addition, hippocampal neurons, RAW 264.7 macrophages and human umbilical vein endothelial cells (HUVECs) were used to exam nitric oxide (NO) production and NO synthase (NOS) gene expression.

**Results:**

*DP*, Hy-*DP* and 5-*u*RCK dose-dependently relaxed isolated rat aortic rings contracted with phenylephrine; however, Hy-*DP* was more effective than *DP*. _L_-NAME and ODQ differentially inhibited Hy-*DP*- and 5-*u*RCK-induced relaxation; both _L_-NAME and ODQ completely blocked 5-*u*RCK-mediated relaxation. Endothelium-denuded aortic ring relaxation was induced much less by 5-*u*RCK than by Hy-*DP*. Therefore, 5-*u*RCK and Hy-*DP* induced vascular relaxation by endothelium-dependent and partially endothelium-dependent mechanisms, respectively. Hy-*DP* and 5-*u*RCK induced eNOS gene expression and NO production in endothelial cells but did not change iNOS/nNOS expression or NO production in macrophages or neuronal cells. Both Hy-*DP* and 5-*u*RCK effectively induced vascular relaxation via similar but slightly different mechanisms. The best effective combination was investigated after mixing Hy-*DP* and 5-*u*RCK at different ratios. The 2:1 Hy-*DP*:5-*u*RCK mixture inhibited ACE, cGMP- and cAMP-dependent phosphodiesterase activity and vascular relaxation better than the other mixtures.

**Conclusion:**

In conclusion, Hy-*DP* and 5-*u*RCK exert antihypertensive effects through different endothelium-dependent or endothelium-independent mechanisms. These findings may greatly help elucidate the mechanisms of clinical efficacy of Hy-*DP*:5-*u*RCK mixtures used for blood pressure regulation.

## Background

Studies on the prevention of hypertension have shown that nutritional intervention may reduce the necessary doses and adverse effects of drugs when used in combination with current pharmacologic treatments [1]. Therefore, nutrition-based approaches are recommended as first-line treatments for the prevention of hypertension in individuals with high-normal blood pressure and as add-on treatments to be used in combination with antihypertensive drugs in patients with hypertension at any stage [2].

Bokbunja refers to Korean black raspberry (*Rubus coreanus* Miq.) fruit and derived products, and is native to Korea, Japan, and China. Unripe *R. coreanus* is a functional food or nutraceutical supplement that is useful for the prevention of noncommunicable diseases, especially cardiovascular diseases (CVDs). We previously reported the effects of a 5% ethanol extract of unripe *R. coreanus* (5-*u*RCK) on CVD-related diseases such as hyperlipidemia and obesity [3–6]. The effects of this extract may reduce the risk for CVDs, including hypertension, atherosclerosis, stroke and myocardial infarction. One of the major active compounds in *R. coreanus* is ellagic acid, which has anti-obesity and antioxidant properties [7, 8]. The unripe fruits of *R. coreanus* are usually used as traditional medicine and might be more therapeutic than the ripe fruits. A recent report revealed that the unripe fruits of *R. coreanus* have a higher concentration of ellagic acid than the ripe fruits, which might be the reason why unripe fruits are traditionally used [9]. Furthermore, our previous study reported that ellagic acid is a major component of 5-*u*RCK [4, 6, 10]. However, information about the antihypertensive effect of 5-*u*RCK is very limited.

*Dendropanax morbiferus* H. Lév., a subtropical tree called *Hwangchil* in Korea due to its golden color lacquer, belongs to the Araliaceae family. It is an endemic species in Korea and is found in the southwestern parts of the country and extracts from its roots and stems are traditionally used to treat migraine headaches, dysmenorrhea, and skin diseases [11]. Biologically active molecules in *D. morbiferus* leaf extract (*DP*), including flavonoid and polyacetylene compounds, have antioxidant, anticancer, antidiabetic and antiatherogenic properties [12–14]. Recently, a report demonstrated that *DP* contains phenolic compounds, including rutin, chlorogenic acid, (+)-catechin, ferulic acid, myricetin, quercetin, and resveratrol, that have anti-inflammatory effects [15]. In our previous study, we suggested quercetin as a marker compound of *D. morbiferus* after analyzing plant parts (fruits, sprouts, leaves, sprigs, and branches), harvest times, and extraction solvents for quality control [16]. In another study, we reported that _L_-arginine and γ-aminobutyric acid (GABA) levels in *DP* were increased by enzymatic hydrolysis and extraction (producing Hy-*DP*) [17]. _L_-arginine is the substrate for nitric oxide (NO) synthesis, which is important for normal endothelial function [18]. GABA-rich products also significantly reduce blood pressure in mildly hypertensive patients [19]. It has been proposed that GABA, one of the depressive neurotransmitters in the central nervous system, plays an important physiological role in the regulation of cardiovascular function [20]. GABA is present in various kinds of common foods, including anaerobically treated tea [21] and fermented foods [22], and the antihypertensive activities of GABA [23] and GABA-containing foods [24] have been reported.

Moreover, we recently reported an antiobesity effect of *DP* [25]. However, information about the antihypertensive effect of *DP* is very limited. Therefore, in this study, the antihypertensive effects of *DP* and Hy-*DP* were investigated in an isolated rat aorta model, and the detailed mechanisms were explored. In addition, the Hy-*DP*/5-*u*RCK combination with the best antihypertensive effect was investigated.

## Methods

### Reagents

N^ω^-nitro-_L_-arginine methyl ester (_L_-NAME), 1H-[1,2,4]oxadiazolo[4,3-a]quinoxalin-1-one (ODQ), _L_-arginine, lipopolysaccharide (LPS; from *Escherichia coli* 0111:B4), phenylephrine hydrochloride (PHE) and angiotensin-converting enzyme (ACE) were purchased from Sigma-Aldrich (St. Louis, MO, USA). Acetylcholine chloride (ACh), glutamic acid and GABA were purchased from Tocris (Ellisville, MO, USA). Dulbecco’s modified Eagle’s medium (DMEM) and fetal bovine serum (FBS) were purchased from Invitrogen, Inc. (Grand Island, NY, USA). All other chemicals were of analytical grade.

### Animals

Specific pathogen-free (SPF) grade healthy male Sprague–Dawley (SD) rats weighing 250 to 300 g each were purchased from Central Lab Animal, Inc. (Seoul, Republic of Korea). Animals were maintained at a constant room temperature of 22 ± 2 °C with a humidity level of 50 ± 5% and with free access to water and food under a 12:12 h light:dark cycle (lights on at 8:00 am). The animals were acclimatized for 4 days before the beginning of the experiments. All efforts were made to minimize animal suffering and to reduce the number of animals used. The experiment was conducted according to the international guidelines for the care and use of laboratory animals [26], and was approved by the institutional animal care and use committee (IACUC) of the Bioresources and Technology (B&Tech) Co., Ltd., Republic of Korea (Approval number: BT-008-2017). When the experiment began, all rats were anesthetized with isoflurane and then sacrificed by cervical dislocation in accordance with the IACUC guidelines; the thoracic aorta of rats was carefully removed.

### Preparation of extracts

The unripe *R. coreanus* fruits (specimen voucher number: BT-URCK001) used in this study were collected (May 2017) in Gochang County (Jeollabuk-do, Republic of Korea) and authenticated by Dr. Kim at B&Tech, Gwangju, South Korea. Extracts of the unripe *R. coreanus* were made using 20 volumes of 5% ethanol at 100 °C for 4 h as described in our previous study [3–6]. The dried leaves of *D. morbiferus* (specimen voucher number: BT-DP001) used in this study were collected (December 2017) in Gangjin County (Jeollanam-do, Republic of Korea) and authenticated by Dr. Kim at B&Tech. *DP* and *Hy-DP* extraction was performed as described in our previous study [17]. Briefly, the dried leaves of *D. morbiferus* were subjected to enzymatic hydrolysis by protease, trypsin, bromelain and papain to increase _L_-arginine and GABA levels. After the leaves were hydrolyzed twice, extraction was performed with purified water at 100 °C for 4 h, and the enzymes were inactivated. Normally, 20.4 g and 27.7 g of dried powder could be obtained from 100 g of unripe *R. coreanus* and *D. morbiferus*, respectively. The Hy-*DP* was then analyzed for the presence of _L_-arginine and GABA using the method described in our previous study [17].

### Ex vivo experiments for measurement of vascular responsiveness

SD-rat thoracic aortas were resected and placed in fresh Krebs’ buffer solution (in mmol/L; NaCl 119, KCl 4.7, CaCl_2_∙2H_2_O 2.5, KH_2_PO_4_ 1.2, MgSO_4_∙7H_2_O 1.2, NaHCO_3_ 25 and glucose 11 at 37 °C) bubbled with 5% CO_2_ and 95% O_2_. The adjacent connective tissues were carefully removed to avoid distention of the vessels and damage to the endothelium. As indicated, the endothelium was removed by rubbing the intimal surfaces of rings with a pair of forceps. The aortas were then cut into 2 mm long rings. In order to minimize the animals used, at least five rings were prepared per rat and the sample sizes usually were 10–25 in our study. The smooth muscle tissue was stabilized in a chamber for 1 h with a resting tension of 2–3 g with saline changes every 20 min. Isometric contractions were recorded using a force-displacement transducer (AD Instruments, Castle Hill, NSW, Australia) under a resting tension of 1.5 g. The rings were contracted again with PHE (10 μM) before construction of a concentration–relaxation curve upon treatment with either ACh or compounds. To determine the NO- or NO-sensitive guanylate cyclase (GC)-mediated relaxation of compounds, the aortic rings were rinsed and exposed to _L_-NAME (10 μM), a NO synthase inhibitor; ODQ (10 μΜ), a NO-sensitive GC inhibitor; or a mixture of _L_-NAME and ODQ for 30 min before induction of steady contraction by PHE. The changes in vascular tension were recorded, and the vasodilation rate (%) was calculated as:

$$ \mathrm{Relaxation}\ \left(\%\right)=\left(\mathrm{maximal}\ \mathrm{contraction}\ \mathrm{by}\ \mathrm{PHE}-\mathrm{tension}\ \mathrm{at}\ \mathrm{the}\ \mathrm{corresponding}\ \mathrm{time}\ \mathrm{after}\ \mathrm{incubation}\ \mathrm{with}\ \mathrm{tested}\ \mathrm{compounds}\right)/\left(\mathrm{maximal}\ \mathrm{contraction}\ \mathrm{by}\ \mathrm{PHE}-\mathrm{basal}\ \mathrm{tension}\right)\times 100\%. $$

### Cell preparation

Cultured hippocampal neurons were prepared using the method described in our previous study [27]. Briefly, the hippocampi were isolated from 16 ~ 18-day-old fetal SD rats and incubated with 0.25% trypsin in Hanks’s Balanced Salt Solution (HBSS) at 37 °C for 20 min. The cells were then mechanically dissociated with fire-polished Pasteur pipettes by trituration and plated at a density of 1 × 10^6^ cells/cm^2^ on poly-_L_-lysine-coated culture dish. The cells were maintained in Neurobasal/B27 medium containing 0.5 mM _L_-glutamine, 25 mM glutamate, 25 mM 2-mercaptoethanol, 100 U/mL penicillin and 100 μg/mL streptomycin under a humidified atmosphere of 95% air and 5% CO_2_ at 37 °C. The cultures were fed twice a week with the same medium without glutamate. Experiments were carried out on neurons after 7–12 days in culture and after the neurons were incubated with 50 μM _L_-glutamate for 6 h as a positive control to induce nNOS.

Murine RAW 264.7 macrophages (40071) were obtained from the Korea Cell Line Bank (KCLB, Seoul, Korea) and cultured in DMEM. To induce an inflammatory state, the cells were grown until 70% confluence was reached and then incubated with 1 μg/mL LPS for 6 h as a positive control to induce iNOS.

HUVECs were obtained from the American Type Culture Collection (ATCC, Manassas, VA, USA). The cells were cultured in medium consisting of modified Kaigen’s F-12 (ATCC) supplemented with 10% FBS, 0.1 mg/mL heparin, and 0.03 mg/mL endothelial cell growth supplement (Upstate, Lake Placid, NY, USA). The cells were grown until 70% confluence was reached and then incubated with 10 μM ACh for 6 h as a positive control to induce eNOS.

### Gene expression analysis

Gene expression in cultured cells was analyzed by RT-PCR, as previously described [28]. Total RNA was extracted from the cultured cells using an easy-BLUE Total RNA Extraction Kit (iNtRON Biotechnology, Seongnam, Republic of Korea) according to the manufacturer’s instructions. To synthesize cDNA, 1 *µ*g of total RNA was mixed with a premixture of oligo (dT) primers and incubated at 45 °C for 60 min. The specific primers that we used in this study were as follows: iNOS, 5′-CAGTTCTGCGCCTTTGCTCAT-3′ (sense) and 5′-GGTGGTGCGGCTGGACTTT-3′ (antisense); eNOS, 5′-GTGTTTGGCCGAGTCCTCACC-3′ (sense) and 5′-CTCCTGCAAGGAAAAGCTCTG-3′ (antisense); and nNOS, 5′-CACATTTGCATGCATGGGCTCGA-3′ (sense) and 5′-CTCTGCAGCGGTATTCATTC-3′ (antisense). Sense (5′-AGGCCGGTGCTGAGTATGTC-3′) and antisense (5′-TGCCTGCTTCACCACCTTCT-3′) primers for glyceraldehyde 3-phosphate dehydrogenase (GAPDH) were used as a control to measure the total RNA content of each sample. Linear amplification range for each gene was tested on the adjusted cDNA. The accumulation of gene transcript was determined by RT-PCR at the 27th cycle. Expression levels were quantified using a gel documentation and analysis system (ChemiDoc XRS+ System, Bio-Rad, Sydney, Australia). A quantitative real-time RT-PCR technique was used to analyze the mRNA expression of eNOS. To normalize mRNA expression, the expression of the housekeeping gene GAPDH was used. The relative mRNA levels were quantified using the ΔΔCt method.

### NO production assay

Various concentrations of 5-*u*RCK and Hy-*DP* were prepared in phenol red-free medium to reduce assay interference by phenol red. Cell culture supernatants were collected after treatment with different compounds for 3 h. NO production was detected spectrophotometrically via measurement of its final stable equimolar degradation products, nitrite (NO^−^_2_) and nitrate (NO^−^_3_), by using nitrate reductase and via measurement of the acid-catalyzed diazotation reaction by using sulfanilamide and naphthyl ethylenediamine (Griess reaction). Total nitrite was quantified after the reduction of all nitrates with nitrate reductase. The nitrite levels in the culture supernatants were within the linear ranges of calibration curves that were generated from a solution of sodium nitrite. The total nitrite concentration was calculated from a standard curve constructed over the linear range of the assay and is expressed in μg/mL.

### Determination of ACE-inhibitory activity

ACE-inhibitory activity was measured according to the method of Holmquist et al. [29] with some modifications. The total volume of 1.22 mL contained 20 μL (20 mU) of commercial ACE (1 U/mL), a 200 μL mixture of different amounts of compounds and 1 mL of 0.5 mM *N*-(3-[2-furyl]acryloyl)-Phe-Gly-Gly). The decrease in absorbance reading at 345 nm (ΔA_inhibition_) was recorded over 5 min at room temperature. Deionized water was used instead of sample solution to obtain a blank reading (ΔA_blank_). ACE activity is expressed as the ACE inhibition (%) and was calculated as follows: [1-ΔA_inhibition_/ΔA_control_] × 100%. The half-maximal inhibitory concentration (IC_50_) was defined as the concentration of sample required to inhibit 50% of ACE activity under these conditions.

### cAMP or cGMP-dependent phosphodiesterase (PDE) activity inhibition assay

The PDE activity inhibition of the compounds was examined using a PDE assay kit (Abcam, Cambridge, MA, USA). Briefly, 10 μL of the compound in distilled water was mixed with 20 μL of 0.5 mM 3′5′-cGMP or 3′5′-cAMP substrate solution, 5 μL of PDE assay buffer, 10 μL of 5 kU/μL 5′-nucleotidase solution, and 5 μL of 4 U/mL PDE solution in each well of 96-well microplates. The mixtures were incubated at 37 °C for 60 min. The absorbance of the mixtures was measured at 620 nm by a microplate reader (EPOCH 2, BioTek, Winooski, VT, USA). The inhibition of PDE activity was calculated by the following equation:

$$ \%\mathrm{inhibition}\ \mathrm{of}\ \mathrm{PDE}\ \mathrm{activity}=\left[{\mathrm{AR}}_{\mathrm{water}}-\left({\mathrm{AR}}_{\mathrm{sample}}-{\mathrm{AC}}_{\mathrm{sample}}\right)/{\mathrm{AR}}_{\mathrm{water}}\right]\times 100, $$

where AR_water_ and AR_sample_ are the absorbances of the mixtures obtained from the reaction of PDEs with distilled water and samples, respectively, and AC_sample_ is the absorbance of the control system (used to determine the phosphate content existing in the compounds).

### Statistical analysis

Best-fit lines were computed for all concentration–response curves using the logistic equation:

$$ \mathrm{y}/{\mathrm{y}}_{\mathrm{max}}=1/\left[1+{\left({k}_{1/2}/\left[\mathrm{A}\right]\right)}^{\mathrm{nH}}\right], $$

where *y*_max_ is the maximal response, *k*_1/2_ is the concentration eliciting the half-maximal response (EC_50_ or IC_50_), [A] is the drug concentration, and *n*_H_ is the Hill coefficient.

The data are presented as the mean and standard error of the mean (SEM) from three independent experiments with replication. The data were statistically evaluated using Student’s *t*-test or two-way analysis of variance (ANOVA) with GraphPad Prism 5 version 5.01 for Windows (GraphPad, Inc., San Diego, California, USA) software programs. Differences between groups were assessed using Duncan’s multiple range tests. Statistical significance was indicated when *p* < 0.05.

## Results

### _L_-arginine and GABA contents of DP, Hy-DP and 5-uRCK

As shown in Table 1, quantitative analysis by HPLC showed that the extracts *DP*, Hy-*DP* and 5-*u*RCK contained 2.61 ± 1.02 mg/g, 17.77 ± 1.36 mg/g and 1.63 ± 0.25 mg/g _L_-arginine, respectively. GABA was also detected by a similar method.

**Table 1:** _L_-Arginine and GABA contents in *DP*, Hy-*DP* and 5-*u*RCK. All results are expressed as the means ± standard deviation of at least three separate experiments. ^**^P < 0.01 and ^***^P < 0.001 vs *DP*

Amino acid	MW	_L_-Arginine and GABA contents (mg/g of extract)		
		***DP***	**Hy-*DP***	**5-*u*RCK**
_**L**_**-Arginine**	174.20	2.61 ± 1.02	17.77 ± 1.36 ^***^	1.63 ± 0.25
**GABA**	103.12	15.53 ± 3.10	27.81 ± 3.78 ^**^	1.09 ± 0.06

### Effects of DP, Hy-DP and 5-uRCK on isolated rat aortic rings precontracted with PHE

As shown in Fig. 1, ACh concentration-dependently caused relaxation in PHE-precontracted (10 μΜ) aortic rings with intact endothelia. Through preliminary screening of *u*RCK extracts prepared by various extraction methods, we found that 5-*u*RCK had the highest vasorelaxant effect (data not shown). In addition, all our previous studies have indicated that 5-*u*RCK has the greatest antiobesity and antihypercholesterolemic effects of all tested *u*RCK extracts [3–6]. As shown in Fig. 1b and g, 5-*u*RCK (EC_50_ value: 1.19 ± 0.06 μg/mL) dose-dependently relaxed endothelium-intact aortic rings precontracted with PHE. As shown in Fig. 1c and d, *DP* (EC_50_ value: 0.55 ± 0.04 μg/mL) and Hy-*DP* (EC_50_ value: 0.57 ± 0.03 μg/mL) also dose-dependently relaxed endothelium-intact aortic rings precontracted with PHE. The maximal relaxant effects of *DP* and 5-*u*RCK on PHE-induced contraction were 78.01 ± 2.86% and 93.84 ± 2.50% at a concentration of 10 μg/mL, respectively. Furthermore, the maximal relaxant effect of Hy-*DP* on PHE-induced contraction was 118.04 ± 6.83% at a concentration of 10 μg/mL. _L_-arginine and GABA, the major components of Hy-*DP*, also showed their own vasodilatory effects. Among them, Hy-*DP* exhibited the most potent vascular relaxant effect.

**Fig. 1:** Effects of *DP*, Hy-*DP* and 5-*u*RCK on thoracic aorta function. Representative traces of vascular relaxant responses induced by ACh (**a**), 5-*u*RCK (**b**), *DP* (**c**) and Hy-*DP* (**d**) in rat thoracic aortae precontracted with 10 μM PHE. Percentages of relaxation in response to increasing concentrations of ACh, _L_-arginine (Arg) and GABA (**e**); *DP* and Hy-*DP* (**f**); and 5-*u*RCK (**g**) in aortic rings from SD rats. The relaxation (%) values (mean ± SEM) are relative to the basal (submaximal) relaxation levels measured before PHE treatment, which were taken to be 100%. ^*^P < 0.05, ^**^P < 0.01 and ^***^P < 0.001 vs *DP*-treated aortae

### Effects of _L_-NAME, ODQ and endothelium denudation on DP-, Hy-DP- and 5-uRCK-induced relaxation in isolated rat aortic rings precontracted with PHE

As shown in Fig. 2a and b, *DP*- and Hy-*DP*-induced relaxation was significantly inhibited by pretreatment with _L_-NAME, ODQ or a mixture of _L_-NAME and ODQ in rat aortic rings with intact endothelia. Moreover, the use of the _L_-NAME and ODQ mixture almost completely inhibited 5-*u*RCK-induced relaxation. Therefore, NO and GC strongly affect the relaxant effect of 5-*u*RCK in an endothelium-dependent manner. Comparison between groups with intact (+E) and denuded (−E) epithelia revealed that the vasodilatory effect induced by *DP* in rings with PHE precontraction was significantly impaired after physical removal of endothelial cells (Fig. 2c), which showed that vasodilation was partially endothelium-dependent. However, Hy-*DP*-induced relaxation in rat aortic preparations was more significantly inhibited (36.69 ± 4.82%) than *DP*-induced relaxation (17.55 ± 7.01%) by denudation of the endothelial layer (Fig. 2d). The data indicate that Hy-*DP* might be responsible for partially endothelium-dependent vasorelaxation. 5-*u*RCK relaxed PHE-induced contractions in +E but not −E aortae (85.06 ± 2.82% inhibition), as shown in Fig. 2c and d. As shown in Fig. 2e, the 5-*u*RCK-induced relaxation response occurred in a dose-dependent manner (E_max_ value: 86.99 ± 3.24), and this relaxation was inhibited by _L_-NAME (E_max_ value: 23.30 ± 3.42), ODQ (E_max_ value: 29.02 ± 2.72) or aortic denudation (E_max_ value: 24.99 ± 2.19). The data indicate that 5-*u*RCK might be responsible for endothelium-dependent vasorelaxation.

**Fig. 2:** Effect of _L_-NAME and ODQ on rat thoracic aorta relaxation induced by 0.3 μg/mL (**a**) and 1 μg/mL (**b**) *DP*, Hy-*DP* and 5-*u*RCK. _L_-NAME, ODQ and a mixture of both (10 μΜ each) were superfused continuously over the strips. (**c**) Vasorelaxant effects of *DP*, Hy-*DP* and 5-*u*RCK in thoracic aortas with denuded endothelia (−E) and intact endothelia (+E). The relaxation (%) values (mean ± SEM) are relative to the basal (submaximal) relaxation levels measured before PHE treatment, which were taken to be 100%. ^NS^*P* > 0.05, ^*^P < 0.05, ^**^P < 0.01 and ^***^P < 0.001 vs *DP*-only-treated aortae; ^##^*P* < 0.01, ^###^*P* < 0.001 vs Hy-*DP*-only-treated aortae; ^$$$^*P* < 0.001 vs _L_-arginine-only-treated aortae; and ^&&&^*P* < 0.001 vs 5-*u*RCK-only-treated aortae. (**d**) Inhibition of the vasorelaxant effects of *DP*, Hy-*DP* and 5-*u*RCK in endothelium-free thoracic aortae precontracted with 10 μM PHE. (**e**) Dose-dependent relaxation (%) induced by 5-*u*RCK in strips of isolated rat thoracic aortic rings with intact endothelia (+E) and denuded endothelia (−E)

### A GABA receptor antagonist suppressed DP- and Hy-DP-induced vasorelaxation

To examine endothelium-independent *DP*- or Hy-*DP*-induced vasorelaxation in greater detail, whether the GABA receptor is involved in *DP*- or Hy-*DP*-induced vasorelaxation was further investigated. As shown in Fig. 3a, 100 μM GABA typically relaxed PHE-induced vasocontraction in endothelial-intact aortae. Pretreatment with bicuculline (a GABA binding site antagonist) did not influence PHE-induced vasocontraction (data not shown), but it suppressed *DP*- or Hy-*DP*-induced vasorelaxation. Likewise, as shown in Fig. 3b and Fig. 3c, *DP*- or Hy-*DP*-induced vasorelaxation was suppressed by pretreatment with flumazenil (a benzodiazepine-binding site antagonist) and picrotoxin (a noncompetitive ionotropic GABA receptor antagonist).

**Fig. 3:** Effects of bicuculline (**a**), flumazenil (**b**) and picrotoxin (**c**) on the relaxation responses induced by *DP* and Hy-*DP* in rat thoracic aortae precontracted with 10 μM PHE. ^***^P < 0.001 vs no blockers

### Effects of Hy-DP and 5-uRCK on NOS gene expression

NOS genes, such as iNOS, nNOS and eNOS, are differentially expressed in response to various stimuli, such as LPS, glutamate and ACh. RT-PCR analysis was performed to determine whether the effects of *DP*, Hy-*DP* and 5-*u*RCK on NO are related to modulation of the expression of NOSs. As shown in Fig. 4a, in LPS-stimulated RAW 264.7 cells, iNOS was strongly expressed. However, iNOS expression was not increased by treatment with *DP*, Hy-*DP* or 5-*u*RCK. Likewise, as shown in Fig. 4b, nNOS expression was not increased by treatment with *DP*, Hy-*DP* or 5-*u*RCK in cultured hippocampal neurons, but nNOS was strongly expressed in glutamate-stimulated cultured hippocampal neurons. We further investigated the effects of *DP*, Hy-*DP* and 5-*u*RCK on eNOS mRNA expression using RT-PCR. eNOS mRNA expression levels were significantly increased in *DP*-, Hy-*DP*- and 5-*u*RCK-stimulated HUVECs (Fig. 4c). Furthermore, eNOS was also strongly expressed in _L_-arginine- and GABA-stimulated HUVECs. eNOS mRNA expression was confirmed by real-time qPCR (Fig. 4d). The eNOS mRNA levels in HUVECs were significantly higher in ACh-treated cells than in control cells and were significantly increased by the *DP*, Hy-*DP* and 5-*u*RCK treatments, except for 0.1 μg/mL *DP* treatment.

**Fig. 4:** Effects of *DP*, Hy-*DP* and 5-*u*RCK on the expression of NOS isoforms at the mRNA level (as assessed by RT-PCR). **a** RT-PCR analysis of iNOS mRNA expression in murine RAW 264.7 macrophages. Activated cultures were stimulated for 6 h with 1 μg/mL LPS or individual extracts before extraction of RNA. **b** RT-PCR analysis of nNOS mRNA expression in cultured rat hippocampal neurons. Activated cultures were stimulated for 6 h with 50 μM _L_-glutamate (Glu) or individual extracts before extraction of RNA. **c** RT-PCR analysis of eNOS mRNA expression in HUVECs. Activated cultures were stimulated for 6 h with 10 μM ACh or individual extracts before extraction of RNA. **d** eNOS mRNA expression was detected by real-time quantitative RT-PCR. ^*^P < 0.05, ^**^P < 0.01 and ^***^P < 0.001 vs the CTL group; NS, not significant

### Hy-DP and 5-uRCK stimulate the production of NO

To further clarify the eNOS-specific expression effects of *DP*, Hy-*DP* and 5-*u*RCK, we compared the amounts of NO produced by RAW 264.7 macrophages, cultured hippocampal neurons and HUVECs in vitro after the different treatments (Fig. 5). NO production was unaffected by both Hy-*DP* and 5-*u*RCK in RAW 264.7 macrophages and cultured hippocampal neurons, whereas exposure to slightly higher concentrations of Hy-*DP* or 5-*u*RCK significantly decreased NO production. Treatment with 30 μM _L_-arginine significantly decreased NO production in RAW 264.7 cells compared with control levels. Furthermore, compared with the control condition, Hy-*DP,* 5-*u*RCK and _L_-arginine treatment significantly decreased NO production in cultured hippocampal neurons. As shown in Fig. 5c, however, HUVEC-mediated release of NO dose-dependently increased after treatment with *DP*, Hy-*DP* and 5-*u*RCK. Culture medium containing supplemental _L_-arginine or GABA significantly increased NO levels in endothelial cells. However, NO production was not further enhanced in the presence of Hy-*DP* compared with *DP* (Fig. 5c).

**Fig. 5:** Effects of *DP*, Hy-*DP* and 5-*u*RCK on NO levels. NO levels in murine RAW 264.7 macrophages, hippocampal neurons, and HUVECs treated with *DP*, Hy-*DP* or 5-*u*RCK. NO production at baseline (control; CTL) and after treatment with 1 μg/mL LPS or individual extracts in murine RAW 264.7 macrophages (**a**), at baseline and after treatment with 50 μM Glu or individual extracts in cultured rat hippocampal neurons (**b**), and at baseline and after treatment with 10 μM ACh or individual extracts in HUVECs (**c**). ^*/#^*P* < 0.05, ^**/##^*P* < 0.01 and ^***/###^*P* < 0.001 vs the CTL group; Symbols refers to the significant difference (* symbol: increase/# symbol: decrease) of treated group to control. NS, not significant

### Combined effects of Hy-DP and 5-uRCK on ACE activity inhibition

As shown in Fig. 6a and b, the effects of different concentrations of *DP*, Hy-*DP* and 5-*u*RCK on ACE activity were examined in vitro. *DP* and 5-*u*RCK both exhibited dose-dependent in vitro ACE inhibition activity, with IC_50_ values of 81.48 ± 0.24 μg/mL and 19.74 ± 0.09 μg/mL, respectively. Hy-*DP* showed greater inhibitory activity (IC_50_ value: 66.70 ± 0.13 μg/mL) than *DP* but far less inhibitory activity than the 2:1 mixture (IC_50_ value: 7.65 ± 0.15 μg/mL). However, ACE activity inhibition was unaffected by all concentrations of both _L_-arginine and GABA (Fig. 6c).

**Fig. 6:** **a**, **b** Inhibitory effects of *DP*, Hy-*DP*, 5-*u*RCK and mixtures of Hy-*DP* and 5-*u*RCK on ACE activity in vitro. Different concentrations and mixture ratios of Hy-*DP* and 5-*u*RCK were added to the reaction mixtures, and ACE inhibition was recorded. ^*^P < 0.05 and ^**^P < 0.01 vs the 1:0 group 10 μg/mL); ^#^*P* < 0.05 and ^##^*P* < 0.01 vs the 1:0 group 30 μg/mL). **d**, **e** Inhibitory effects of *DP*, Hy-*DP*, 5-*u*RCK and mixtures of Hy-*DP* and 5-*u*RCK on cGMP-dependent PDE activity in vitro. Different concentrations and mixture ratios of Hy-*DP* and 5-*u*RCK were added to the reaction mixtures, and cGMP-dependent PDE inhibition was recorded. **g**, **h** Inhibitory effects of *DP*, Hy-*DP*, 5-*u*RCK and mixtures of Hy-*DP* and 5-*u*RCK on cAMP-dependent PDE activity in vitro. Different concentrations and mixture ratios of Hy-*DP* and 5-*u*RCK were added to the reaction mixtures, and cAMP-dependent PDE inhibition was recorded. ^**^P < 0.01 vs the 1:0 group 1 μg/mL); ^#^*P* < 0.05 vs the 1:0 group 3 μg/mL). **c**, **f**, **i** Inhibitory effects of GABA and _L_-arginine (Arg) on ACE- and cGMP−/cAMP-dependent PDE activity in vitro

### Combined effects of Hy-DP and 5-uRCK on cGMP-dependent PDE inhibition

The cGMP-dependent PDE-inhibitory effects of *DP*, Hy-*DP* and 5-*u*RCK were tested and compared with those of 3-isobutyl-1-methylxanthine (IBMX), a PDE inhibitor drug (positive control). The IC_50_ value of IBMX was 24.2 ± 1.14 μM (data not shown). The highest cGMP-dependent PDE inhibition percentage was observed for the 2:1 mixture (10 μg/mL) at 95.50 ± 0.92% (Fig. 6d and e). This mixture yielded an IC_50_ value of cGMP-dependent PDE inhibition of 0.34 ± 0.04 μg/mL. However, as Fig. 6f shows, no significant changes in PDE inhibition were observed after treatment with varying doses of _L_-arginine and GABA.

### Combined effects of Hy-DP and 5-uRCK on cAMP-dependent PDE inhibition

The activity of PDEs, which are known to hydrolyze cAMP into inactive 5′ nucleotide monophosphates (5′-adenosine monophosphate [AMP]) [30], was not significantly altered by treatment with varying doses of _L_-arginine and GABA (Fig. 6i). However, the highest cAMP-dependent PDE inhibition percentage was observed for the 2:1 mixture (10 μg/mL) at 89.64 ± 2.70% (Fig. 6g and h). This mixture yielded an IC_50_ value of cAMP-dependent PDE inhibition of 1.68 ± 0.25 μg/mL.

### Combined effects of Hy-DP and 5-uRCK on isolated rat aortic rings precontracted with PHE

As shown in Fig. 7a and b, the 1:1 mixture (EC_50_ value: 2.68 ± 0.11 μg/mL) dose-dependently relaxed endothelium-intact aortic rings precontracted with PHE. The 2:1 mixture (EC_50_ value: 0.39 ± 0.02 μg/mL) also dose-dependently relaxed endothelium-intact aortic rings precontracted with PHE. The maximal relaxant effects of the 1:1 mixture and 2:1 mixture on PHE-induced contraction were 65.58 ± 3.97% and 130.71 ± 4.77% at a concentration of 10 μg/mL, respectively. Therefore, the 2:1 mixture exhibited the most potent vascular relaxant effect.

**Fig. 7:** Relaxation in response to increasing concentrations of *DP*, Hy-*DP*, 5-*u*RCK and Hy-*DP*/5-*u*RCK mixtures in rat aortic rings. The concentration–response curves show the relaxation effects of *DP*, Hy-*DP*, 5-*u*RCK and mixtures of Hy-*DP* and 5-*u*RCK on rat thoracic aortae precontracted with PHE in the presence of functional endothelium (**a**). Summary of the EC_50_ values of different extracts with regard to the relaxation of endothelium-intact aortic rings precontracted with PHE (**b**). All values are expressed as the means ± SEMs

## Discussion

This present study demonstrated, for the first time, that Hy-*DP* and 5-*u*RCK induced significant endothelium-dependent and endothelium-independent relaxation in PHE-precontracted aortic rings. To investigate the involvement of NO, the aortic rings were pretreated with _L_-NAME. Pretreatment with _L_-NAME completely abolished the vasorelaxation induced by 5-*u*RCK; however, it did not completely abolish the vasorelaxation induced by Hy-*DP*. Interestingly, the relaxation induced by 5-*u*RCK, but not that induced by Hy-*DP*, was completely abolished in denuded aortic rings. These results indicated that 5-*u*RCK exhibited an endothelium-dependent vasodilator effect, while Hy-*DP* exhibited a partially endothelium-dependent vasodilator effect. Additionally, Hy-*DP* and 5-*u*RCK significantly increased nitrate/nitrite levels and eNOS expression in vitro, thereby increasing NO bioavailability. Although _L_-NAME is a nonspecific inhibitor of all three NOS isozymes, eNOS plays a major role in the development and maintenance of hypertension. This study addressed the specific effects of Hy-*DP* and 5-*u*RCK on the neuronal and inducible NOS isozymes. The results confirmed that Hy-*DP* and 5-*u*RCK did not affect the expression of neuronal or inducible NOS but specifically increased the expression of eNOS. Interestingly, combined treatment with Hy-*DP* and 5-*u*RCK induced increased relaxation in PHE-precontracted aortic rings, producing additive effects compared with treatment with either Hy-*DP* of 5-*u*RCK alone. In particular, the most significant effect was observed when Hy-*DP* and 5-*u*RCK were mixed at a 2:1 ratio.

It is known that endothelial cells generate NO from _L_-arginine via the catalytic action of eNOS [31]. Intracellular _L_-arginine concentrations usually remain in the range of 0.8–2.0 mM, implying that the endothelium is always saturated with _L_-arginine as a substrate for constitutively active eNOS-mediated NO synthesis. However, as the external supply of _L_-arginine decreases, _L_-arginine transcellular transport becomes the rate-limiting step in NO production. Therefore, NO released by endothelial cells is regarded as an important regulator of vascular function. We have previously established an enzymatic hydrolysis extraction method to amplify the _L_-arginine content in *DP* and Hy-*DP* [17]. The results showed that _L_-arginine contained in Hy-*DP* could ameliorate vascular dysfunction caused by deficiency of _L_-arginine. However, the exact molecular mechanisms of Hy-*DP-* and 5-*u*RCK-activated _L_-arginine transport remain to be further studied.

The integrity of the vascular endothelium is pivotal for health, and the cardiovascular protective activity of the endothelium depends on its capacity to generate NO [32]. It is also known that inhibition of eNOS activity impacts the constitutive release of NO in vessel walls. The results of the present study with regard to both intact endothelia and eNOS activity showed that both Hy-*DP* and 5-*u*RCK mediated vasodilation at clinically useful doses. Therefore, we are conducting additional studies to identify effective concentration ranges and elucidate the detailed mechanisms using hypertension animal models, such as the spontaneously hypertensive rat (SHR) model and the 1 kidney-1 clip (1 K-1C) Goldblatt rat model of hypertension.

eNOS is one of the isoforms of the NOS family responsible for NO production in endothelial cells [33]. The activity of eNOS is highly regulated by its interaction with various proteins, such as calmodulin (CaM), heat shock proteins, the B2 receptor, caveolin and dynamin-2 [34]. Phosphorylation by various protein kinases at serine residues and, to a lesser extent, threonine and tyrosine residues has been recently identified to be an important regulator of eNOS activity [34]. Phosphorylation at Ser1177 is carried out by protein kinase A (PKA) or GMP- and AMP-dependent kinases [34]. Although this study did not elucidate the detailed mechanisms involved in the phosphorylation of these proteins, Hy-*DP* and 5-*u*RCK were found to selectively increase eNOS expression. Therefore, we will follow up with this study to determine the effects of Hy-*DP* and 5-*u*RCK on the phosphorylation of eNOS and its related proteins.

The ability of Hy-*DP* to induce relaxation in the presence of _L_-NAME or in the denuded aortic rings indicates the involvement of constituents that act through different vascular mechanisms, independent of the endothelium. We tested the hypotheses that GABA contained in Hy-*DP* exhibits a vasorelaxant effect and that Hy-*DP* regulates ACE- or PDE enzyme activity.

Previous studies have reported that a single oral administration of GABA (0.5 mg/kg) significantly lowers systolic blood pressure in SHRs [23] but not in normotensive rats and that the antihypertensive activity of GABA is dose-dependent at doses ranging from 0.05 to 5 mg/kg in SHRs [24]. Since 100 mg of Hy-*DP* contains 2.8 mg of GABA, as estimated from the HPLC data, we found that Hy-*DP* contains a high enough concentration of GABA to decrease blood pressure in SHRs.

Food products that inhibit ACE activity in vitro have been considered ideal candidates for alleviation of hypertension [35]. Moreover, one mechanism that has been proposed to explain the antihypertensive effect of the extract is the inhibitory effect of the extract on ACE. This present study demonstrated that Hy-*DP* exhibited considerably stronger ACE-inhibitory activity (IC_50_ = 66.70 μg/mL) than *DP* (IC_50_ = 81.48 μg/mL). However, _L_-arginine and GABA did not show ACE-inhibitory activity. Furthermore, the cGMP-dependent PDE-inhibitory activity observed for Hy-*DP* (IC_50_ = 0.40 μg/mL) was considerably stronger than that of *DP* (IC_50_ = 0.73 μg/mL). However, _L_-arginine and GABA did not show ACE- or PDE-inhibitory activity. Therefore, the ACE- and PDE-inhibitory activity of *DP* and Hy-*DP* may be due to various flavonoids, such as quercetin. According to previous reports, flavonoids such as quercetin-2-*O*-α-6-caffeoyl-glycosyl-β-1,2-rhamnoside (IC_50_ = 158.9 μM), quercetin-3-*O*-α-6-p-coumaroyl-glycosyl-β-1,2-rhamnoside (IC_50_ = 351.6 μM), quercetin-3-*O*-β-glucopyranoside (IC_50_ = 708.8 μM) and quercetin-3-*O*-α-arabinopyranoside (IC_50_ = 320 μM), have strong ACE-inhibitory activity [36, 37]. Furthermore, many flavonoid-rich plants have been reported to exert ACE-inhibitory effects both in vitro and in vivo [38, 39]. Researchers have even suggested that there might be an association between the consumption of flavonoid-rich foods and reductions in blood pressure. As in the case of ACE, the importance of flavonoid compounds for preservation of cardiovascular function and the links between flavonoid components and the NO/cGMP pathway have been emphasized [36]. However, changes in flavonoid content during the enzymatic hydrolysis extraction of *DP* were not identified. Therefore, we need to clarify these findings in further research. We also intend to further study ACE-inhibitory activity and the levels of plasma endothelin-1 in hypertensive animal models such as the SHR model. A further possible mechanism of the antihypertensive effects of Hy-*DP* and 5-*u*RCK may be related to the pronounced PDE-inhibitory activity of these extracts. Reductions in NO synthesis or increases in NO degradation lead to decreases in cGMP formation, which promote vasoconstriction responses, platelet adhesion and proliferation of vascular smooth muscle cells, thus favoring vascular hypertrophy and occlusive vascular disease [40]. PDEs compose a class of enzymes that are capable of cleaving phosphodiester bonds in both cAMP and cGMP, which are important intracellular messengers that stimulate vascular smooth muscle relaxation. Orallo et al. [41] reported that the clear vasorelaxant effects of naringenin, a natural flavonoid, on rat aortic smooth muscle are probably mediated by increases in cytosolic cAMP and cGMP concentrations. As observed for the ACE-inhibitory effects, the increased PDE-inhibitory effects of Hy-*DP* are expected to be due to changes in flavonoid content that occur during the enzymatic hydrolysis step of Hy-DP production.

The cytotoxicity of extracts may be one factor involved in vascular endothelial-independent responses. We have tested and reported the cytotoxicity of *DP* and 5-*u*RCK extracts in various cells through similar studies. As a result, we have not observed any cytotoxicity of these extracts up to 300 μg/mL in 3 T3-L1 cells [5, 6, 21], HepG2 cells [3, 4, 42], human gastric epithelial cell [43], mouse melanoma cells [44] and rat primary hepatocytes [45]. Although this study did not provide direct cytotoxicity results, it is expected that there will be no cytotoxicity according to the results of our previous reports. Therefore, in the next study, it is necessary to study the direct effect on the cytotoxicity of the extract by separating vascular endothelial and muscle cells.

## Conclusions

The main finding of the present study was that the extracts Hy-*DP* and 5-*u*RCK exert vasorelaxant effects through slightly different endothelium-dependent or endothelium-independent mechanisms. The vasorelaxant effects of Hy-*DP* and 5-*u*RCK may be associated with increases in eNOS gene expression and inhibition of ACE and PDE activity. The vasorelaxant effect of Hy-*DP* might be due mostly to the effects of _L_-arginine and GABA and partially to the effects of polyphenols, which have vasodilatory activity. Interestingly, combined treatment with Hy-*DP* and 5-*u*RCK was more effective than treatment with Hy-*DP* or 5-*u*RCK alone. Collectively, these findings suggest that a mixture of Hy-*DP* and 5-*u*RCK could be used for prevention of or as an adjuvant therapy for hypertension. However, more studies are required to evaluate the detailed mechanisms in experimental animal models of hypertension and to determine the safety and efficacy of such a mixture in clinical conditions in humans.

## Data Availability

All data and analyses in the current study are available from the corresponding author upon reasonable request.

## Abbreviations

ACE: Angiotensin-converting enzyme
ACh: Acetylcholine chloride
cAMP: Cyclic 3′,5′-adenosine monophosphate
cGMP: Cyclic 3′,5′-guanosine monophosphate
CVD: Cardiovascular disease
*DP*: *Dendropanax morbiferus* H. Léveille extract
eNOS: Endothelial nitric oxide synthase
EC_50_: Half maximal effective concentration
GABA: γ-aminobutyric acid
GAPDH: Glyceraldehyde 3-phosphate dehydrogenase
GC: Guanylate cyclase
HUVEC: Human umbilical vein endothelial cell
Hy-*DP*: Enzymatically hydrolyzed *Dendropanax morbiferus* H. Léveille extract
IC_50_: Half maximal inhibitory concentration
iNOS: Inducible nitric oxide synthase
_L_-NAME: N^ω^-nitro-_L_-arginine methyl ester
NO: Nitric oxide
NOS: Nitric oxide synthase
nNOS: Neuronal nitric oxide synthase
ODQ: 1H-[1, 2, 4] oxadiazolo [4,3-a]quinoxalin-1-one
PDE: Phosphodiesterase
PHE: Phenylephrine hydrochloride
5-*u*RCK: 5% unripe *Rubus coreanus* Miquel ethanol extract
